# Methane-Rich Saline Counteracts Cholestasis-Induced Liver Damage via Regulating the TLR4/NF-*κ*B/NLRP3 Inflammasome Pathway

**DOI:** 10.1155/2019/6565283

**Published:** 2019-11-18

**Authors:** Zeyu Li, Dongdong Chen, Yifan Jia, Yang Feng, Cong Wang, Yingmu Tong, Ruixia Cui, Kai Qu, Chang Liu, Jingyao Zhang

**Affiliations:** ^1^Department of Hepatobiliary Surgery, The First Affiliated Hospital of Xi'an Jiaotong University, Xi'an, Shaanxi 710061, China; ^2^Department of the First General Surgery, Gansu Provincial Hospital, Lanzhou, Gansu 730000, China; ^3^Department of Immunology, Shaanxi University of Chinese Medicine, Xianyang, Shaanxi 712046, China; ^4^Department of ICU, The First Affiliated Hospital of Xi'an Jiaotong University, Xi'an, Shaanxi 710061, China; ^5^Department of SICU, The First Affiliated Hospital of Xi'an Jiaotong University, Xi'an, Shaanxi 710061, China

## Abstract

Cholestatic liver injury, due to obstruction of the biliary tract or genetic defects, is often accompanied by progressive inflammation and liver fibrosis. Methane-rich saline (MRS) has anti-inflammatory properties. However, whether MRS can provide protective effect in cholestatic liver injury is still unclear. In this study, Sprague-Dawley rats received bile duct ligation (BDL) to generate a cholestatic model followed by MRS treatment (10 mL/kg, ip treatment) every 12 h after the operation to explore the potential protective mechanism of MRS in cholestatic liver injury. We found that MRS effectively improved liver function, alleviated liver pathological damage, and localized infiltration of inflammatory cells. MRS treatment decreased the expression of hepatic fibrosis-associated proteins to alleviate liver fibrosis. Furthermore, MRS treatment suppressed the TLR4/NF-*κ*B pathway and further reduced the levels of proinflammatory factors. Downregulation of NF-*κ*B subsequently reduced the NLRP3 expression to inhibit pyroptosis. Our data indicated that methane treatment prevented cholestatic liver injury via anti-inflammatory properties that involved the TLR4/NF-*κ*B/NLRP3 signaling pathway.

## 1. Introduction

Due to obstruction of the biliary tract or genetic defects, cholestasis is a widespread clinical liver disease. Cholestatic liver injury occurs in many diseases, such as cholestasis during pregnancy, primary sclerosing cholangitis (PSC), drug-induced cholestasis liver disease, and cholestasis liver disease caused by various types of viral hepatitis [1]. The accumulation of highly toxic bile acid causes cholestatic liver damage, hepatic inflammation, proliferation of hepatic stellate cells (HSCs), and ultimately hepatic fibrosis, cirrhosis, and death [2]. However, the detailed mechanism of the initiation of inflammation induced by toxic bile acid is still unknown [3].

Toll-like receptors (TLRs) are a key member of the cellular transmembrane receptors and pathogenic membrane recognition receptors in the innate immunity. TLRs activate the immune response by recognizing invasive pathogens and promote the release of inflammatory cytokines via interactions with NF-*κ*B. TLR4 recognizes the LPS leading to the activation of NF-*κ*B, translocating NF-*κ*B to the nucleus, and secreting the proinflammatory cytokines, such as tumor necrosis factor-*α* (TNF-*α*), interleukin-6 (IL-6), and interleukin-1*β* (IL-1*β*) [4]. Moreover, NF-*κ*B can further promote the conversion of IL-18 and IL-1*β* precursors to mature IL-18 and IL-1*β*, which play key roles in NLRP3-mediated pyroptosis [5]. During the inflammation, NLRP3, activated by TLRs, promotes the caspase-1 precursors to mature caspase-1 which further induce the release of the IL-1*β* and IL-18. This process is protective during the initial inflammation. However, when IL-1*β* and IL-18 are continually released and accumulated in the cell, it causes pyroptosis, tissue damage, and organ dysfunction [6]. Therefore, the hepatic damage during obstructive cholestasis might be related with the NLRP3 pathway.

Methane is a small organic-reducing molecule of the simplest alkane and has obtained increasing attention, particularly for disease treatment. Recently, the study of the MRS on sepsis-induced acute kidney injury has shown that MRS can inhibit the CHOP signaling pathway to provide a positive effect [7]. Methane can also alleviate intestinal ischemia/reperfusion (IR) injury in a rat model [8]. In addition, MRS upregulates PI3K/signaling pathway expression, which alleviates liver injury induced by carbon tetrachloride [9]. Boros et al. found that exogenous inhalation of methane had anti-inflammatory effects on ischemia-reperfusion-induced oxidative and nitrosative stress [10]. Thus, methane is a type of novel and nontoxic organic gas that possesses substantial antioxidative, anti-inflammatory, and antiapoptotic properties. In this study, MRS was prepared and used to investigate its protective effect on cholestasis-induced liver damage and to explore the specific underlying mechanisms to provide a novel treatment of cholestasis.

## 2. Materials and Methods

### 2.1. Rats and Bile Duct Ligation

Male Sprague-Dawley (SD) rats were kept under controlled conditions (23~25°C, 12 h light/dark cycle) for 1 week before experiment. The 4% chloral hydrate was used to anesthetize rats, and the cholestasis-associated hepatic damage was induced by bile duct ligation performance [11]. Midline laparotomy, dissection of the common bile duct, double-ligation with silk suture, and cutting of the bile duct between the ligatures were routinely performed on rats. The sham and MRS control groups underwent an operation just to expose the bile duct without ligating. After that, the abdomen was closed in layers.

### 2.2. Experimental Design

Male SD rats were assigned into four groups randomly (*n* = 10 per group): sham control group, MRS control group, BDL+NS group, and BDL+MRS group. Rats in the sham and MRS control groups underwent a sham laparotomy operation, and 10 mL/kg normal saline (NS)/methane-rich saline (MRS) was respectively administered every 12 h after BDL for seven days. Rats in the BDL+NS and BDL+MRS groups underwent a BDL operation, and 10 mL/kg NS/MRS was respectively administered every 12 h after BDL for seven days. Seven days after BDL operation, rats were euthanized to collect the blood and tissue samples which were stored at -80°C for further biochemical analysis.

### 2.3. The Preparation of Methane

The methane saline was produced as previously described which was freshly prepared 1 day before experiments to ensure a steady concentration [12]. The concentration of MRS was 1.2-1.5 mmol/L which was detected by using gas chromatography as the previous study [13].

### 2.4. Histologic Analysis

Hematoxylin and eosin (H&E) staining and Masson staining were adopted to detect the pathological changes. Liver tissues were fixed with 10% formalin solution and embedded in paraffin. 4 *μ*m serial sections were used to stain with H&E and Masson's trichrome. Liver histologic change was observed and assessed by two researchers in a double-blinded way through a light microscope. Histological scores were guided by previous experiments [14].

### 2.5. Inflammatory Cytokine Assay

Seven days after BDL operation, the blood samples were collected and serum samples were centrifuged to measure the TNF-*α*, IL-6, and IL-1*β* levels using ELISA kits (Dakewe, China).

### 2.6. Western Blot Assay

Seven days after the BDL operation, the expression of *α*-SMA, TGF-*β*1, collagen I, TLR4, Myd88, p65, p-p65, NLRP3, caspase-1, and IL-1*β* was measured using western blotting with antibodies purchased from San Ying Biotechnology (China), CST (USA), Abcam (USA), Beyotime Biotechnology (China), and Abmart (China). The total protein in liver tissues was extracted by RIPA lysis buffer at 14000*g* for 15 min at 4°C. 15 *μ*g protein in each samples was separated by SDS-PAGE and transferred onto PVDF membranes which were blocked and incubated overnight at 4°C with specific primary antibodies (NLRP3 1 : 1500, *α*-SMA 1 : 500, and others 1 : 100). Then, the washed membranes were incubated with the secondary antibody (1 : 1000) for 1 h at room temperature. Finally, the protein bands were visualized using the chemiluminescent analysis system. Bands were analyzed and quantified using ImageJ software.

### 2.7. Immunohistochemical Analysis

Immunohistochemistry was used to detect the F4/80, TGF-*β*1, collagen I, *α*-SMA, NLRP3, and caspase-1 expression in the liver tissues. The antibodies were purchased from San Ying Biotechnology (China), Abcam (USA), and Beyotime Biotechnology (China). Briefly, the liver samples were fixed and sliced as described before. The sections were deparaffinized, were rehydrated with serial gradient ethanol, and blocked endogenous peroxidase activity with 3% hydrogen peroxide. The sections were incubated overnight at 4°C with primary antibodies against F4/80 (1 : 200), *α*-SMA (1 : 100), TGF-*β*1 (1 : 400), collagen I (1 : 400), NLRP3 (1 : 100), and caspase-1 (1 : 150). The washed sections were incubated with peroxidase-conjugated anti-rabbit antibody at room temperature for 40 min. Finally, the slides were stained with diaminobenzidine tetrahydrochloride (DAB), counterstained with hematoxylin and mounted for microscopic examination.

### 2.8. Immunofluorescence Staining

After collection, the liver samples were fixed and sliced as described before. Immunofluorescence for TLR4 and NF-*κ*B expression was performed as previously described [15]. The antibodies were purchased from Wuhan Bioss (China), Servicebio (China), and Abcam (USA). The primary Ab TLR4 (1 : 400) and p65 (1 : 200) were incubated overnight at 4°C and amplified with the secondary Ab at 37°C for 60 min. The slides were incubated with 4′-6-diamidino-2-phenylindole (DAPI). The fluorescence microscope was used to observe the sections. ImageJ software was used to measure the quantification of fluorescence intensity.

### 2.9. Statistical Analysis

Data were presented as the mean ± SD. One-way ANOVA followed by SNK tests was used to determine significant differences for comparisons among 3 or more groups. All statistical analysis was performed by using Prism 7 (GraphPad Software Inc.). *p* < 0.05 was considered statistically significant.

## 3. Results

### 3.1. MRS Treatment Improved Liver Function in DBL Rats

Massive inflammatory cell infiltration was observed in H&E staining of the liver tissues 7 days after BDL in the BDL+NS group (Figure 1(a)). And the necrotic tissues and the infiltration of inflammatory cells in the liver were significantly alleviated by MRS treatment. Compared with those in the sham control group and MRS control group rats, the liver injury score increased markedly at 7 days in the BDL+NS group (Figures 1(b) and 1(c)). MRS treatment significantly reduced the above change (*p* < 0.01). The levels of TBIL, ALT, and AST were significantly increased after BDL, which was consistent with the histologic data (Figures 1(d)–1(f)). The levels of these liver injury indicators 7 days after BDL were alleviated by MRS treatment (*p* < 0.05).

### 3.2. MRS Treatment Downregulates Inflammatory Responses after BDL

Inflammation is one of the main factors in liver damage in cholestatic diseases. To investigate the macrophage infiltration, F4/80 (a macrophage marker) immunostaining was performed. IHC staining of the liver showed a large amount of macrophage infiltration 7 days after BDL compared with the sham control group and the MRS control group (Figure 2(a)). MRS treatment effectively reduced infiltration of liver macrophages during cholestasis (*p* < 0.05) (Figure 2(b)). Excessive proinflammatory factors (TNF-*α* and IL-6) aggravate cholestatic liver injury [11]. The serum levels of TNF-*α* and IL-6 significantly increased by 13- and 3.2-fold, respectively, 7 days after BDL (Figures 2(c) and 2(d)). The serum levels of TNF-*α* and IL-6 were significantly decreased by 42.0% and 23.0% with MRS treatment.

### 3.3. MRS Treatment Alleviated Liver Fibrosis Formation in BDL Rats

Then, we investigated whether MRS treatment could decrease the expression of *α*-SMA, TGF-*β*1, and collagen I. As shown in Figure 3(a), western blot assay demonstrated that *α*-SMA, TGF-*β*1, and collagen I were highly expressed in the BDL+NS group 7 days after BDL operation. MRS treatment effectively reduces the expression of *α*-SMA, TGF-*β*1, and collagen I. Quantification of the relative protein expression verified these findings (Figures 3(b)–3(d)). Compared with the BDL+NS group, IHC staining has also shown a less expression of *α*-SMA, TGF-*β*1, and collagen I in the BDL+MRS group (Figures 3(e)–3(h)). Masson's trichrome staining analysis also supported this result above, which showed significant reduction in levels of liver fibrosis in the BDL+MRS group compared with the BDL+NS group (Figures 4(a) and 4(b)). These data suggest that MRS treatment not only inhibits inflammation but also inhibits the activation of KCs, further mitigating fibrosis formation in BDL rats.

### 3.4. MRS Treatment Downregulated TLR4/NF-*κ*B Signal Pathway Expression

The TLR4/NF-*κ*B signal pathway could promote and amplify the inflammatory response during inflammation [16]. Western blot was used to examine the levels of TLR4/NF-*κ*B proteins. Compared with the sham and MRS control groups, the western blot assay in the BDL+NS group revealed a dramatically increased expression of TLR4/NF-*κ*B. However, the levels of the TLR4/NF-*κ*B signal pathway in the BDL+MRS group were profoundly decreased by MRS treatment. These findings were verified by quantification analysis of the relative protein expression levels (Figures 5(b)–5(d)). To further confirm this result, we measured TLR4 and p65 expression via immunofluorescence staining (Figures 5(e)–5(h)). Compared with the sham and MRS control groups, TLR4-positive cells in the BDL+NS group showed a significantly increasing trend, and the trend was inhibited by MRS treatment. In addition, the p65-positive cells also increased in the BDL+NS group. Administration of MRS significantly reduced p65-positive cells in the liver. Therefore, we concluded that MRS inhibited TLR4/NF-*κ*B signal pathway activation to reduce the generation of proinflammatory cytokines.

### 3.5. MRS Treatment Inhibited NLRP3 Inflammasome Activation and Reduced Pyroptosis

The activation of NF-*κ*B upregulates the expression of NLRP3 protein, which subsequently promotes more production of IL-1*β* and eventually leads to pyroptosis [17]. NLRP3 inflammasome activation is correlated with liver fibrosis during BDL [18]. Next, we investigated whether MRS treatment could inhibit the activation of NLRP3 inflammasome. According to the result of western blot, the levels of NLRP3/caspase-1/IL-1*β* expression significantly increased in the BDL+NS group compared with the sham and MRS control groups (Figure 6(a)). MRS treatment reduces this increase. These findings were verified by quantification analysis of the relative protein expression levels (Figures 6(b)–6(d)). In addition, we also measured NLRP3 and caspase-1 expression via immunohistochemistry staining (Figures 6(e)–6(g)). NLRP3 and caspase-1 expression dramatically increased in BDL+NS rats compared with the sham and MRS control groups. However, MRS treatment attenuated the increase in the BDL+MRS group. Finally, we measured IL-1*β* expression in serum via ELISA (Figure 6(h)). Similarly, IL-1*β* expression was increased in the BDL+NS group in contrast to the sham and MRS control groups. MRS treatment decreased IL-1*β* levels in serum. These results suggested that MRS reduced the liver fibrosis in a cholestatic rat model through inhibition of pyroptosis by downregulating the expression of the NLRP3 inflammasome signaling pathway.

## 4. Discussion

Biliary obstruction is a life-threatening disease that causes excessive inflammatory response and liver damage, eventually leading to liver fibrosis and increased mortality [19]. During cholestasis, excessive inflammatory responses can activate the TLR4 signaling pathway, which promotes NF-*κ*B activation to secrete more proinflammatory cytokines, like TNF-*α* and IL-6, to aggravate inflammatory damage and liver fibrosis. Moreover, the activation of NF-*κ*B can further upregulate the expression of the NLRP3 inflammasome, leading to pyroptosis [20]. However, there is still no good method for the treatment of cholestasis liver damage clinically.

Methane possesses antioxidative, anti-inflammatory, and antiapoptotic properties, which have been proved through a septic mouse model [13]. Furthermore, methane exhibited good effects on sepsis-induced mice kidney injury, intestinal IR injury, and liver IRI [8, 12]. However, there is no evidence suggesting that MRS possesses protective effects on cholestatic liver fibrosis. Liver mitochondria are critically involved in cholestasis-induced cellular damage. Hepatocyte mitochondrial damage produces excessive oxygen free radicals, which induce activation of the NLRP3 inflammasome [21]. Strifler et al. have showed that methane can improve mitochondrial respiration [22]. Meszaros et al. demonstrated that mitochondria are targets of methane [23]. Considering this characteristic, we hypothesize that MRS can inhibit inflammation and mitochondrial damage-induced pyroptosis to protect against liver damage in a cholestatic rat model.

To determine the effect of MRS on BDL-induced cholestasis, we performed in vivo experiments. We generated a cholestasis rat model via bile duct ligation (BDL) and found that BDL-induced cholestasis induced rat liver tissue damage and liver fibrosis. After the BDL operation, H&E and Masson's trichrome staining showed significant macrophage infiltration, bile duct necrosis, and liver fibrosis in rats. MRS treatment effectively improved liver pathological damage in rats. The levels of TBIL, ALT, and AST were significantly decreased in BDL rats treated with MRS.

The inflammatory response plays a key role in the pathogenesis of cholestasis. TNF-*α* and IL-6, regulated by NF-*κ*B, are involved in every stage of immune response and inflammatory response [24]. In addition, excessive production of TNF-*α* and IL-6 also leads to a decrease in bile flow, which further leads to cholestasis [25]. Meanwhile, cholestasis can also aggravate the inflammatory response in liver tissue. Studies have shown that MRS treatment can reduce inflammatory responses [10]. In our study, the levels of proinflammatory cytokines (TNF-*α* and IL-6) were decreased by MRS treatment, suggesting that MRS may attenuate liver injury in cholestasis via the reduced inflammatory response and macrophage infiltration.

In addition, massive activation of Kupffer cells also contributes to BDL-induced inflammation in the liver injury. KCs express TLR4 and are activated during cholestasis. Activated TLR4 stimulates the activation of NF-*κ*B and further results in the upregulation of the inflammatory response [26]. Conversely, cholestasis-induced liver damage in mice is effectively reduced by blocking TLR4 signaling or NF-*κ*B activation [11]. Our study showed that MRS treatment could inhibit cholestasis-induced activation of TLR4/NF-*κ*B. Cholestasis activates NF-*κ*B to mediate NLRP3 inflammasome expression. The NLRP3 inflammasome, a multiprotein complex, promotes the conversion of caspase-1 precursor to mature caspase-1 during inflammation. The mature caspase-1 further drives inflammatory response by converting pro-IL-1*β* to IL-1*β*, subsequently inducing pyroptosis. NLRP3 inflammasome activation subsequently aggravates liver fibrosis and cholestasis [27]. In our study, the BDL operation significantly increased NLRP3 inflammasome signal pathway expression, resulting in liver fibrosis. MRS treatment could reduce activation of the NLRP3 inflammasome signal pathway and inhibit pyroptosis, thus reducing liver fibrosis in BDL rats.

In conclusion, the present study showed that methane treatment could prevent cholestatic liver injury mainly inhibiting the inflammation and decreasing the pyroptosis through downregulation of the TLR4/NF-*κ*B/NLRP3/caspase-1/IL-1*β* signal pathway. These findings bring a promising prospect that methane treatment may be a feasible and complementary method for the treatment of cholestatic liver injury.

## Figures and Tables

**Figure 1:** MRS alleviated tissue damage and organ dysfunction in the livers of BDL rats. Rats were treated by intraperitoneal administration (10 mL/kg) of MRS for 7 days after BDL. Liver tissues and blood samples were collected 7 days after the BDL operation. (a) H&E staining (scale bars: 100 *μ*m and 50 *μ*m). (b) Necrotic areas. (c) Histological scores. (d–f) Serum levels of TBIL, ALT, and AST (*n* = 10. Data are shown as the mean ± SD. ^∗^*p* < 0.05 versus the sham control group; ^#^*p* < 0.01 versus the sham control group; ^€^*p* < 0.05 versus the MRS control group; ^$^*p* < 0.01 versus the MRS control group; ^&^*p* < 0.05 versus the BDL+NS group; *^γ^p* < 0.01 versus the BDL+NS group).

**Figure 2:** Methane-rich saline alleviated inflammatory responses in BDL-induced liver damage. Rats were treated via intraperitoneal administration (10 mL/kg) of MRS for 7 days after BDL. (a) F4/80 immunohistochemical staining was used for the detection of macrophage infiltration. (b) Positive rate of F4/80 cells. The levels of (c) TNF-*α* and (d) IL-6 were measured with commercial ELISA kits. MRS treatment reduced serum TNF-*α* and IL-6 concentrations (*n* = 10, scale bars: 20 *μ*m. Data are shown as the mean ± SD. ^∗^*p* < 0.05 versus the sham control group; ^#^*p* < 0.01 versus the sham control group; ^€^*p* < 0.05 versus the MRS control group; ^$^*p* < 0.01 versus the MRS control group; ^&^*p* < 0.05 versus the BDL+NS group; *^γ^p* < 0.01 versus the BDL+NS group).

**Figure 3:** Methane-rich saline inhibited the expression of hepatic fibrosis-associated protein in BDL rats. MRS treatment in rats was achieved by intraperitoneal administration (10 mL/kg) for 7 days after BDL. (a) Immunoblot assays of *α*-SMA, TGF-*β*1, and collagen I. Relative densities of (b) *α*-SMA, (c) TGF-*β*1, and (d) collagen I. (e) Immunohistochemical staining of *α*-SMA, TGF-*β*1, and collagen I. The percentage of (f–h) *α*-SMA, TGF-*β*1, and collagen I. (*n* = 10, scale bars: 20 *μ*m. Data are shown as the mean ± SD. ^∗^*p* < 0.05 versus the sham control group; ^#^*p* < 0.01 versus the sham control group; ^€^*p* < 0.05 versus the MRS control group; ^$^*p* < 0.01 versus the MRS control group; ^&^*p* < 0.05 versus the BDL+NS group; *^γ^p* < 0.01 versus the BDL+NS group).

**Figure 4:** Methane-rich saline repressed liver fibrosis formation in BDL rats. MRS treatment in rats was achieved by intraperitoneal administration (10 mL/kg) for 7 days after BDL. (a) Masson's trichrome staining (scale bars: 100 *μ*m and 50 *μ*m). (b) The densitometry data of Masson's trichrome staining (*n* = 10. Data are shown as the mean ± SD. ^∗^*p* < 0.05 versus the sham control group; ^#^*p* < 0.01 versus the sham control group; ^€^*p* < 0.05 versus the MRS control group; ^$^*p* < 0.01 versus the MRS control group; ^&^*p* < 0.05 versus the BDL+NS group; *^γ^p* < 0.01 versus the BDL+NS group).

**Figure 5:** Methane-rich saline downregulated the expression of the TLR/NF-*κ*B signaling pathway. MRS treatment in rats was achieved by intraperitoneal administration (10 mL/kg) for 7 days after BDL. (a) Immunoblot assays of TLR4, Myd88, and NF-*κ*B (p65). Relative densities of (b–d) TLR4, Myd88, and NF-*κ*B (p65). (e) Immunofluorescence staining of TLR4. (f) The percentage of TLR4-positive cells. (g) Immunofluorescence staining of NF-*κ*B (p65). (h) The percentage of NF-*κ*B (p65)-positive cells. (*n* = 10, scale bars: 25 *μ*m. Data are shown as the mean ± SD. ^∗^*p* < 0.05 versus the sham control group; ^#^*p* < 0.01 versus the sham control group; ^€^*p* < 0.05 versus the MRS control group; ^$^*p* < 0.01 versus the MRS control group; ^&^*p* < 0.05 versus the BDL+NS group; *^γ^p* < 0.01 versus the BDL+NS group).

**Figure 6:** Methane-rich saline reduced pyroptosis via inhibiting inflammasome signaling pathway activation. MRS treatment in rats was achieved by intraperitoneal administration (10 mL/kg) for 7 days after BDL. (a) Immunoblot assays of NLRP3, caspase-1, and IL-1*β*. Relative densities of (b–d) NLRP3, caspase-1, and IL-1*β*. (e) Immunohistochemical staining of NLRP3 and caspase-1 (scale bars: 20 *μ*m). The percentage of (f, g) NLRP3 and caspase-1. (h) IL-1*β* serum levels (*n* = 10. Data are shown as the mean ± SD. ^∗^*p* < 0.05 versus the sham control group; ^#^*p* < 0.01 versus the sham control group; ^€^*p* < 0.05 versus the MRS control group; ^$^*p* < 0.01 versus the MRS control group; ^&^*p* < 0.05 versus the BDL+NS group; *^γ^p* < 0.01 versus the BDL+NS group).

## Data Availability

The data related to mouse model data, serum cytokine levels, histological staining, and western blot images used to support the findings of this study are available from the corresponding authors upon request.

## Abbreviations

MRS: Methane-rich saline
BDL: Bile duct ligation
Sham control group: Sham-operated group
MRS control group: Sham-operated with MRS treatment group
BDL+NS group: Normal saline treatment group with bile duct ligation
BDL+MRS group: Methane-rich saline treatment with bile duct ligation
TBIL: Total bilirubin
AST: Aspartate aminotransferase
ALT: Alanine aminotransferase
TLR4: Toll-like receptor 4
NF-*κ*B: Nuclear factor-kappa B
NLRP3: NOD-like receptor protein 3
*α*-SMA: Alpha smooth muscle actin
TGF-*β*1: Transforming growth factor beta 1.
